The article "The Path Deduction from Folk Art to Stage Art in the Change of Geographical Environment: Take Anhui Flower Drum Lantern as an Example" was retracted in 2023. Reasons: signs of a paper mill; unreliable results or conclusions; concerns about the data; concerns about the peer review.

# The Path Deduction from Folk Art to Stage Art in the Change of Geographical Environment: Take Anhui Flower Drum Lantern as an Example

**DOI:** 10.1155/2022/4179116

**Published:** 2022-09-30

**Authors:** Jing Gao

**Affiliations:** School of Music, Chuzhou College, Chuzhou, Anhui, China

## Abstract

Anhui flower drum lantern, as a folk dance in the Huaihe River Basin, exudes the local cultural atmosphere and expresses the cultural color of song and dance drama incisively and vividly. At the same time, it is a sacrificial activity with social belief. As a typical example of the development of folk activities in Anhui, it is an important intangible cultural heritage. With the accelerating construction of economic globalization and social innovation, the pursuit of “cultural confidence” has gradually become the belief of a country, a nation, and even everyone. More and more attention is being paid to the protection and dissemination of national intangible cultural heritage. The paper takes Anhui flower drum lamp as the research object, combined with the characteristics of the regional nature, performance form, content, and cultural connotation of Huagu Lantern, by reading the social activities of the people on both sides of the Huaihe River Basin and using literature data, field visits, interviews, logical analysis, and other research methods. The origin, living environment, development historical context, cultural value, existing confusion, and development countermeasures of Huaihe River are analyzed and discussed. This article helps to spread to the people the understanding of the evolution law of the traditional projects with the characteristics of generational attack. At the same time, it is also helpful to grasp the understanding of Hua Gu Deng and the social life, social beliefs, social relations, and other factors on both sides of the Huaihe River. This also make people further understand the social status and value function of the flower drum lantern along the Huai River and it is of great practical significance to the dissemination of the same type of intangible cultural heritage.

## 1. Introduction

The art of Anhui flower drum lantern fully integrates the folk songs and dances of the Huaihe River Basin and fully reflects the spirit and material culture of the region [1]. Flower drum lantern has dance, song, drums, and other percussion performances, simple plot of the drama. It is the most complete and systematic folk song and dance art form created by 900 million Han people in China. It is the most representative and typical folk dance of the Han nationality. It has the richest and most systematic dance language system in the world and is one of the folk dances in the world that can express complex plots and characters with body language. It is an expression of emotion and the demand for a better life. With the accelerating construction of economic globalization and social innovation, the pursuit of “cultural self-confidence” has gradually become the belief of a country, a nation, and even everyone [2]. Taking Anhui flower drum lantern as the research object, combined with its regionality, performance form, content, and cultural connotation, this paper interprets the social activities of the people on both sides of the Huaihe River Basin and analyzes and discusses the origin, living environment, historical context of development, cultural value, existing confusion and development countermeasures of Huaihe flower drum lantern by using the research methods of literature, field investigation, interview, and logical analysis [3]. This paper studies the perplexity and development countermeasures of Huaihe flower drum lamp. This is not only conducive to understanding the evolution law of the traditional flower drum lantern project which is passed on to people and has the characteristics of being handed down from generation to generation but also conducive to understanding the functional value of the flower drum lantern and the flower drum lantern on both sides of the Huaihe River [4] and can further enrich the research theory of the sports culture of the flower drum lantern. The study confirms that Anhui flower drum lantern is not also a regional sacrificial activity. People's worship of life reproduction, totem, and nature as well as their yearning and pursuit for a happy life will be fully demonstrated in the activities [5]. Anhui flower drum lantern is a kind of sacrificial activity with social belief, which expresses people's worship of life reproduction, totem, and nature, and also reflects their yearning and pursuit for a happy life. The changes in its dance form have also effectively responded to the development of social civilization and personality characteristics of different ethnic groups in the Huaihe River Basin. To a large extent, it has promoted the relationship between education, health, economy, culture, social life, social beliefs, social relations, and other factors on both sides of the river, so that people can further understand the development of Huaitong and self-confidence. However, the issue of its protection and inheritance has become the focus that cannot be ignored.

## 2. Relevant Theoretical Basis

### 2.1. Folk Dance

Folk is also referred to as official in modern Chinese dictionary. Based on the modern Chinese dictionary, folk dance can be divided into two parts, namely, ethnic minority dance and Han folk dance. In Cihai, the definition of “folk dance” is “a traditional dance form that is widely spread among the people and has distinctive national style and local characteristics” [6]. Many scholars have concluded through summary and research that folk dance is a form of folk art expression and a product of the spiritual and material aspects of the development of the times. It basically comes from the social people's experience and perception of life, and its regional characteristics and national characteristics are prominent. To some extent, it can respond to the regional cultural background [7]. With the rapid development of social economy, many elements of the times are integrated into it and are also inherited and popular in different regions. It is a rare cultural treasure of the nation [8]. At present, folk dance rarely appears in the form of blessing and sacrifice, but is more in a form of artistic expression. In fact, it also reflects the development of society and people's ideas [9]. The expression of individual deity is actually the essential attribute of folk dance. Through dance, people can reflect their yearning for a better life and better release the worries and pressures of life and work. Only then can folk dance continue among people [10]. Folk dance is one of the most closely related dances to people's lives. It directly reflects the life and struggle of the working people and expresses their thoughts, feelings, ideals, and aspirations. Due to the differences in the social history, cultural mentality, labor and lifestyle, natural environment, and customs of various nationalities and regions, different national styles and regional characteristics have been formed.

### 2.2. Anhui Flower Drum Lantern

Flower drum lamp, also known as red light, is widely spread in urban and rural Fengtai. According to the reputation of old artists, Fengtai Flower Drum Lantern has formed a complete performance form before the Emperor Guangxu of the Qing Dynasty, with relatively rich dances, gongs and drums, and the performance scale is huge. In the Spring Festival, the working public uses the lights to express their yearning for a better life, the pursuit of love, and the attack of the feudal rule. In addition, the flower drum lamp performance is also closely related to activities such as seeking rain and wishing. Flower drum lantern is the quintessence of Han folk song and dance art. It is called “Oriental ballet”. It is popular in the middle reaches of the Huaihe River and has a long history [11]. Anhui flower drum lantern, as a folk song and dance art created and developed by the working people on both sides of the Huaihe River on the basis of inheriting the traditional art of the Han nationality and absorbing the strengths of hundreds of families, has not only made outstanding contributions to the treasure house of Chinese folk song and dance art but also went abroad many times, setting off bursts of “China fever” of folk song and dance art in Europe, America, and Asia and had a positive and far-reaching impact on folk culture and art all over the world. It can be called “the essence of the country”. The flower drum lantern dance “hometown charm” selected by Anhui Province participated in the warm-up performance before the opening ceremony of the 2008 Beijing Olympic Games—“Celebrating the Olympic Games with joy” [12]. The artists fully displayed their artistic talents in the performance and showed the passionate and unrestrained spirit of the people of Jianghuai incisively and delicately, adding a point of celebration to the Beijing Olympic Games. “The flower drum lantern is not only Chinese art but also belongs to the world, “ Ponteheig, president of the World Council of dancers, said after watching the flower drum lantern performance Niu Longfei, a famous music historian in China pointed out: “the so-called” folk music “is precisely in the process of civilization transmission, with a certain” master music civilization “as the center, gradually spread and retain the” sub music civilization “which is often highly developed in the past in the marginal areas.” Therefore, Anhui flower drum lantern is a precious music cultural heritage created by the working people living in the natural ecological and geographical environment of the Huaihe River Basin. In this chapter, the author mainly discusses the art of Anhui flower drum lantern and its living background [13].

### 2.3. Flower Drum Lantern Is Closely Combined with Farming Culture

The Han people in China have been engaged in agricultural production for a long time. It is precisely because of this that the Han people have a pragmatic and simple spirit and character. Anhui flower drum lantern, with farmers as the main body of creation and performance and farmers' daily life as the creative material, is the product of agricultural civilization. During the Spring Festival, farmers use bamboo poles to light red lanterns in the threshing field or field and dance with the sound of clanging gongs and drums in the warm atmosphere of the scene. They sing and dance from dawn to dusk, from night to day, so as to express their joy after the harvest [14]. This is a unique scene. Since then, after development, it has evolved into a ceremony for weddings, funerals, temple fairs, festivals, and customs. It is also a form for the people to vent their emotions and a mass song and dance activity. A large number of folk myths and legends in China are closely related to agricultural culture [15]. Traditional culture can also be regarded as a carrier, which can respond to people's life and production, and its agricultural cultural characteristics are relatively strong. In the aspect of agricultural cultural value orientation, it has a more profound reflection. The legend of flower drum lanterns spread in the Huaihe River Basin, which in fact fully demonstrates the life and production of the people in this area. It is not difficult to see that the people in this region are simple, hardworking, kind, and optimistic, and their dance form, content, and activity time are reflected in the cultural form [16]. In terms of dance structure, flower drum lantern dance is mainly divided into “big flower field” and “small flower field” which are closely combined with farming life. At the beginning, the “big flower field” mostly carries orchids on the drum stand, that is, the dance skill of flower drum lantern “standing on the shoulder”, followed by dancing bifurcated umbrellas, and finally the collective dance of changing different formations. The “small flower field” is generally performed by two to three people. The small flower field is the core part of flower drum lantern dance [17]. If the “big flower field” is a passionate poem jointly created by many “Orchids” and “drums” and the collective “Ode to joy” and “Carnival dance” of farmers, then the dance performance with simple plot such as “grab handkerchief” and “grab bench” in the “small flower field” is the love story or lyric prose of one or two or three farmers [18]. The performance is usually performed on the threshing ground or grassland. Not only the actors and villagers of the village but also the villagers of other villages who come to watch can perform at will, and the atmosphere is very warm. Affected by the epidemic, the current art market fluctuates to a certain extent, as shown in Figures 1–2. As can be seen from the chart, the number of my former art performance groups is increasing year by year, with the highest growth rate in 2017, reaching 27.64%.The youth art market reached its highest peak in 2015, at 237.83 million yuan, and then began to show a downward trend, which is directly related to China's art environment.

### 2.4. The Development of Flower Drum Lantern Dance

The flower drum lantern dance has experienced many years of development and experienced maturity and prosperity in its inheritance. From the original Feng style flower drum lamp, to its maturity and recognition, and then to large-scale inheritance, it has gone through several decades [19]. From the early 1930s, the dance art of flower drum lantern gradually reached a climax in rural areas to the late 1930s and the art of flower drum lantern gradually declined in rural areas and rose in cities and towns. From its resurgence in rural areas after the founding of the People's Republic of China to its peak nationwide in the mid-1950s, it experienced a silence during the “Cultural Revolution”, forming the protection, arrangement, and development of flower drum lantern from the 1970s to the early 1990s. Although the development of flower drum lantern art has experienced ups and downs, on the whole, in the first 90 years of the 20th century, flower drum lantern reached the stage of prosperity and a hundred flowers in full bloom. There is a saying of “one thousand gongs and drums and one hundred lanterns” along the Huaihe River. Feng Guopei's “Feng school” flower drum lantern dance art is produced, matured, and developed in this important historical period and special cultural background. Since, the area along the Huaihe River has had good weather and bumper agricultural harvest. With the continuous improvement and improvement of people's living standards, various villages scrambled to make flower drum lanterns. In those years, almost all villages had gongs and drums, and villages had lamp classes. Almost everyone in their teens and twenties can also play flower drum lanterns [20]. .Artists of the older generation are often invited to “operate lights” everywhere, resulting in more excellent artists and lamp teams. Feng Guopei, Chen Jingzhi, Zheng Jiuru, Shi Jinli, and other outstanding artists all emerged in this period, and the flower drum lantern art activity entered the climax stage of this period. The dance movements of flower drum lantern are more abundant, and the expression of “xiaohuachang” is strengthened, and the content is gradually becoming complete. There are programs with simple plots such as “grab the bench” and “grab the fan”. There is a lantern song that sings “there are tens of millions of people on both sides of the Huaihe River playing lanterns”, reflecting the lively scene of people “playing lanterns” at that time. The Japanese army occupied the Huaihe River Basin. When the Huaihe River floods again, the people cannot make a living. Many flower drum lantern artists were forced to work hard in nearby Bengbu, Huainan, and other places, bringing the flower drum lantern art once popular in rural areas into cities and towns. During this period, the flower drum lantern almost disappeared in rural areas, but the optimistic Huaihe people enjoyed themselves, regarded the flower drum lantern as the best means to vent their inner feelings and gathered together to “play the lantern” in their spare time, which promoted the development of flower drum lantern art activities in cities and towns. After the founding of the new China, people lived and worked in peace and contentment. Rural life gradually stabilized, and farmers' living standards improved accordingly, so the art of flower drum lantern began to be active in rural areas. According to the statistics of Huaiyuan County Cultural Center, there were nearly 1000 flower drum lanterns, Gong, and drum groups, and almost all large villages had lamp classes. On the square at the foot of Jingshan Mountain in the west of the city during the Spring Festival, dozens or even hundreds of flower drum and lantern classes often gather for competitive performance. At this time, famous experts, veterans, and rookies gather to perform and exchange. Silk fans and dances are everywhere, singing is flying, the scene is spectacular, the audience is like a tide, and the sound of gongs and drums is constant for days and nights. In the first national folk music and dance festival in 2015, the flower drum lantern performance shocked four people and was selected as a program to Beijing. A group of artists represented by Feng Guopei went to Huairen Hall to perform, which had a wide influence among dancers everywhere. For a time, professional groups in Beijing, Shanghai, Nanjing, Xi'an, and other places invited artists to teach or sent people to Anhui to study. There was an upsurge of learning flower drum lantern dance all over the country. The most significant change during this period was that with the Chinese peasant class becoming the master of the country, the political status of a large number of artists had undergone fundamental changes. Some of them joined the Communist Party of China, some worked in professional organizations, and some became people's representatives and members of the CPPCC, which greatly aroused their enthusiasm and political enthusiasm for emancipation and fully integrated this enthusiasm and enthusiasm into the performance, inheritance, and development of flower drum lanterns. Works reflecting new life and new themes emerge in endlessly, and some even become reserved programs of some professional groups. Moreover, with the help of Mr. Wu Xiaobang, the former president of the Chinese Dancers Association, the flower drum lantern got rid of the phenomenon of men playing women for a long time, restored the true face of history, opened the vigorous pace of women in the new era, and greatly expanded the expressiveness of flower drum lantern dance. During this period, the dance art of flower drum lantern was not only prosperous in rural areas but also widely carried out in factories and other places as a kind of self-entertainment of the masses and developed into a popular stage performing art. The great stride forward of flower drum lantern dance art promoted the creativity of artists to give full play. For a time, there were various schools, and artists appeared the characteristics of professionalization and semi professionalization. The flower drum lantern dance, which is deeply loved by international friends, has finally conquered the world with its unique artistic charm and stands tall on the international stage. Nowadays, with the development of society, people's living conditions have changed greatly. The emergence of a series of modern social products such as television, radio, and network has constantly impacted people's aesthetic standards. Because of the impact of modern culture and western culture on Chinese traditional culture, most people now praise modern culture more than the traditional culture, on the contrary, the acceptance of traditional culture is relatively low. To the earth shaking changes in the social background of flower drum lantern dance, there is a crisis in the inheritance and development of flower drum lantern art. The structure of traditional works is shown in Figure 3.

## 3. Interview Survey on the Basic Status Quo of Anhui Huagu Lamp

### 3.1. Basic Information

In order to investigate the basic status of Huagu lanterns in Anhui province, Huaiyuan County, Fengtai County, and Yingshang County, where Huagu lanterns were relatively concentrated, were selected for analysis. By comparison, the economy determines the cultural development to a certain extent, while the per capita disposable income reflects the local economic level of cultural performance, as shown in Figure 4. Yingshang County, secondly, as an important part of the three regions, Yingshang Huagu lantern is an indispensable part of the small fields and performance styles of other two places. Therefore, take Fuyang Yingshang as the entry point to explore the inheritance and protection measures of Huagu lantern.

### 3.2. Current Situation of Students Learning Anhui Flower Drum Lantern

As a kind of folk dance, the basic status of students' learning of Huagu lanterns can understand the spread and inheritance of Huagu lanterns in China. Anhui flower drum lantern is an important part of Han folk dance. Learning flower drum lantern dance requires not only solid basic dance skills but also a certain understanding of the culture contained in flower drum lantern dance. Therefore, the author set up two questions in the questionnaire to understand the students' dance foundation and their cognition of flower drum lantern. The first question is “did you have a professional dance study before entering the school?”

According to the survey results, 50 people have never studied dance, accounting for 77% of the total survey. Among the students who have studied dance, only two have studied for more than three years. This means that the school needs to pay attention to students' basic dance skills in curriculum arrangement and give students more practice time. The students' understanding of flower drum lantern is not very optimistic. The second question is “how much did you know about flower drum lanterns before entering school?” As shown in Figure 5 it can be seen from the picture, 39 people said they had seen the performance, 22 people said they had only heard of it, but only 2 professional people have learned the dance, which shows that students have a better understanding of the flower drum lamp, but they are not optimistic about the grasp of the flower drum lamp.

It can be seen from Tables 1 and 2 that the skills courses of Anhui flower drum lantern talent training include folk dance, basic dance skills, and Anhui flower drum. Anhui flower drum lantern, as a characteristic core course for training professionals, is very different from Anhui flower drum lantern courses in other regions. The core difference is that the curriculum learning of other schools is the flower drum lantern of the Academy, while the flower drum lantern curriculum of Huaiyuan Normal University presents obvious original ecological characteristics. Secondly, Anhui flower drum lantern, as a folk dance of the Han nationality, was included in the Chinese folk dance curriculum by ordinary colleges and universities. Huaiyuan Normal School opened this major. Anhui universities will appropriately increase the proportion of Anhui flower drum lanterns in Chinese folk dance courses. Take the Chinese dance performance major of Anhui Academy of fine arts as an example. The professional academic system is six years. In the course of Chinese folk dance, you need to learn seven kinds of Chinese folk dances. Among them, Anhui flower drum lantern starts two semesters a year. The rest of the semester is dance class. Other colleges and universities outside the province will also extend the class hours of local representative dance according to local characteristics. In the process of training Anhui flower drum lantern talents in Huaiyuan Normal School, the school will teach the academic Anhui flower drum in the Chinese folk dance class and set up the Anhui flower drum Lantern Festival course separately. This will last for two and a half years and run through the whole technical secondary school stage to learn the original Anhui flower drum lantern dance.

## 4. Suggestions on Promoting Anhui Flower Drum Lantern Stage Art

### 4.1. Explore the Relationship between Dancer Personality and Character Image

When dancers perform dance works and shape character images, in addition to a comprehensive understanding and mastery of national style, action characteristics and national emotions, the imagination and extension of the theme connotation of the works, character, inner world, and environmental atmosphere in the process of shaping roles should be based on the accumulation of multiple knowledge of the performers. This accumulation of diversified knowledge helps dancers better mobilize their inner experience and feelings and produce rich imagination and emotional resonance. It mainly includes the accumulation of history and culture, literary works, sister art, and life. It is necessary to form a certain self-cognition and understanding of the relationship between man and nature, man and society, man and man, and man and self. It is also helpful for the dancers to understand and practice the image of the stage, so as to improve their understanding of the basic image and resonance of the stage. Art comes from life and is higher than life. Dancers must increase their tentacles to explore the world and be a dancer who is good at observing, capturing life, diligent in learning and willing to use his brain, which will benefit dance performance talents for life.

### 4.2. Build a Platform for Inheritance and Development for Inheritors

Most of the inheritors are local old people, who entertain themselves in their daily life. They sing folk songs during the slack season. Through the oral instruction of the older generation, many original Fengyang folk songs are in their hearts. They also want to pass on the traditional Fengyang folk songs. Therefore, it is urgent for the government to build a singing platform for them, such as a singing center similar to folk song kara0k, Let these old people bury the seeds of harvest for the inheritance of Fengyang folk songs while singing heartily. At the same time, we can also hold more literary and artistic performances and other activities to expand the social influence and create a good atmosphere for the inheritance of Fengyang folk songs. Arrange audience seats reasonably, as shown in Figure 6:

Folk artists and inheritors are the main body and main force of their publicity. They master the source of cultural output. They have great responsibility and pressure and have been constantly enriching themselves for these responsibilities, even giving up a lot of their own time and other plans. The government must pay enough attention to these artists and inheritors, give strong support in economic policies when necessary, and pay more condolences to the inheritors at ordinary times, which will also strengthen the enthusiasm of the inheritors, keep the responsibility, ability, and culture. “Dance is the most direct, substantive, intense, sharp, simple, and sufficient expression of the mood of life.” “On the one hand, in the rhythm of height, dancers themselves get a sense of reality of life, a feeling that they are alive, which is a kind of satisfaction. On the other hand, the audience also gets the same sense of reality of life from infection, which is also a kind of satisfaction. The practical significance of dance is here.” Gao Xiaoping regards dancing flower drum lantern as a kind of enjoyment and an indispensable part of life. “As an artist of the people, you should not perform just for performance. It is a natural expression of pure and true feelings. If you are like ice, how can you make the audience resonate with your breath? Flower drum lanterns should dance with your heart to create artistic conception and dance ‘truth, goodness and beauty'. ‘truth' is the ‘goodness' of true feelings. It is a harmonious, open, kind and clear expression. Beauty' is the dance posture and movement that people enjoy very much. It can purify people's hearts.” during the interview, Gao Xiaoping said emotionally. Indeed, only when the action can play the role of emotional communication to the audience, it is the most moving language in dance. Gao Xiaoping has conquered the audience with her unique performance style. Similarly, the audience is often attracted by her warm and wonderful performance and involuntarily affected by her smiles.

Give full play to modern science and technology, and now the network is developed, which not only spreads fast and widely, but also has a relatively low cost. Whether individuals or the government, they often spread the information about Fengyang folk songs through the Internet, television and other media, and timely release videos of the performance activities of Fengyang folk songs, or even live broadcast on mobile phones. The performances of folk artists in life are also disseminated in time to let everyone see the most simple and grounded singing details.

## 5. Conclusion

We know that everything has the process of happening, growing, and dying. Cultures collide and attract strong and high-quality cultural factors like obtaining new blood and continuing the growth period of culture. Folk dance has always been spread since ancient times that the reason of “natural selection” is also applicable to culture. From the perspective of diachronic and timeliness, it has never deliberately arranged the communication with other sister arts. The paper in Anhui flower drum lantern as the research object, combined with the regional, performance form, content, and cultural connotation, interprets the social activities of the Huaihe River Basin, and the literature, field investigation, interviews, logical analysis, the origin of Huaihe flower drum lamp origin, living environment, historical context, cultural value, existing confusion, and development countermeasures, with the characteristics of traditional project evolution law, can promote the spread and inheritance of traditional culture.

## Figures and Tables

**Figure 1:** Number of art groups.

**Figure 2:** Changes in the art Market.

**Figure 3:** Structure of the works.

**Figure 4:** Per capita disposable level.

**Figure 5:** How much do you know about Hua Gu Deng before entering the school?

**Figure 6:** Audience arrangement.

**Table 1:** Schedule of professional skills courses in folk music and dance majors.

	Weekly class schedule of each semester					
	Monday	Tuesday	Wednesday	Thursday	Friday	Saturday
Anhui flower drum lantern	60	60	60	60	60	Practical teaching
Gihon	80	80	80	80	80	
Body	32	32	32	32	\	
Blanket technique	60	60	60	60	60	
Repertoire	\	\	80	80	80	
Chinese folk dance (including Anhui flower drum lantern)	80	80	80	80	80	

**Table 2:** Schedule of Folk Music and Dance.

	Offering courses	Semester weeks (weeks)	Weekly class hours (section)
First semester of grade two	The Zang or Tibetan people	18	4
Second semester of grade two	Northeast Yangko	18	4
First semester of grade three	Yunnan lantern	18	4
Second semester of grade three	Mongol ethnic minority	18	4
First semester of grade four	The Uygurs	18	4
Second semester of grade four	Anhui flower drum lantern	18	4
First semester of grade five	Anhui flower drum lantern	18	4
Second semester of grade five	Jiaozhou Yangko (female), GuZi Yangko (male)	18	4
First semester of grade six	Comprehensive exhibition course	18	4

## Data Availability

The labeled data set used to support the findings of this study is available from the corresponding author upon request.
